# Sequence-Based Appraisal of the Genes Encoding Neck and Carbohydrate Recognition Domain of Conglutinin in Blackbuck (*Antilope cervicapra*) and Goat (*Capra hircus*)

**DOI:** 10.1155/2014/389150

**Published:** 2014-06-16

**Authors:** Sasmita Barik, Chandra Mohan Sidappa, Mohini Saini, Ramesh Doreswamy, Asit Das, Anil K. Sharma, Praveen K. Gupta

**Affiliations:** ^1^CWL, Indian Veterinary Research Institute, Izatnagar, Uttar Pradesh 243 122, India; ^2^Department of Physiology and Biochemistry, Hassan Veterinary College, KVAFSU, Bidar, Karnataka 585401, India; ^3^Animal Biotechnology Division, IVRI, Izatnagar, Uttar Pradesh 243 122, India

## Abstract

Conglutinin, a collagenous C-type lectin, acts as soluble pattern recognition receptor (PRR) in recognition of pathogens. In the present study, genes encoding neck and carbohydrate recognition domain (NCRD) of conglutinin in goat and blackbuck were amplified, cloned, and sequenced. The obtained 488 bp ORFs encoding NCRD were submitted to NCBI with accession numbers KC505182 and KC505183. Both nucleotide and predicted amino acid sequences were analysed with sequences of other ruminants retrieved from NCBI GenBank using DNAstar and Megalign5.2 software. Sequence analysis revealed maximum similarity of blackbuck sequence with wild ruminants like nilgai and buffalo, whereas goat sequence displayed maximum similarity with sheep sequence at both nucleotide and amino acid level. Phylogenetic analysis further indicated clear divergence of wild ruminants from the domestic ruminants in separate clusters. The predicted secondary structures of NCRD protein in goat and blackbuck using SWISSMODEL ProtParam online software were found to possess 6 beta-sheets and 3 alpha-helices which are identical to the result obtained in case of sheep, cattle, buffalo, and nilgai. However, quaternary structure in goat, sheep, and cattle was found to differ from that of buffalo, nilgai, and blackbuck, suggesting a probable variation in the efficiency of antimicrobial activity among wild and domestic ruminants.

## 1. Introduction

Conglutinin, a calcium dependent, collagenous protein of serum, is synthesized from liver [1–4]. It is a member of collectin superfamily [3] having characteristic C-type lectin domain (CTLD). The protein is grouped along with mannan-binding lectin (MBL), lung surfactant protein A (SP-A), lung surfactant protein D (SP-D), collectin liver 1 (CLL1), collectin placenta 1 (CL-P1), collectin 43 kDa (CL-43), and collectin 46 kDa (CL-46). Initially conglutinin was detected in cattle as a serum component, capable of agglutinating erythrocytes opsonized with antibodies and complement [5]. It was thought to be confined to bovines but recent studies revealed reactivity of antiserum rose against bovine conglutinin towards serum protein in other nonruminants [6] and invertebrates [7] as well. The gene encoding conglutinin is located on the bovine chromosome 28q1.8 position [2, 8–11] with other collectin groups of proteins. Functionally active dodecameric form [4] is a tetramer giving cruciform like appearance similar to SP-D, CL-43, and CL-46. The basic monomeric unit consists of N-terminal cysteine-rich domain, a collagen domain, a coiled-coil neck domain, and C-terminal globular carbohydrate recognition domain (CRD). Bovine conglutinin cDNA was first reported to be amplified as 912 bp from liver cDNA library [1]. The complete 1519 bp cDNA encoding bovine conglutinin from liver was cloned and characterized later, which is found to possess an open reading frame of 1116 bp encoding a polypeptide of 371 amino acids, out of which 20 constitute the signal sequence. The mature peptide is found to consist of 351 amino acids [2] with 25 residues at the N-terminal end forming the noncollagenous cysteine-rich domain followed by a collagenous domain of 171 residues with 55 Gly-X-Y repeats interrupted twice, followed by a short segment of coiled-coil neck domain in continuation with 155-residue-long globular C-terminal end referred to as the carbohydrate recognition domain (CRDs) [12, 13].

The protein displays wide spectrum of antimicrobial activities [14] by binding to surface glycan residues on microorganisms either directly or via iC3b protein [15]. Conglutinin binds microorganisms through its lectin domain in a calcium dependent manner and brings their agglutination. Sugar bound conglutinin is also capable of stimulating the reactive oxygen species [16] in various phagocytic cells of immune system that helps in destruction and ultimately clearance of the pathogen from the body [17]. Thus, it serves as an innate immune marker [18] in the form of soluble pattern recognition receptors (PRR) committed to detect the specific pathogen associated molecular pattern (PAMP).

Blackbuck (*Antilope cervicapra*), a wild antelope which belongs to order Artiodactyla of family Bovidae, is a near threatened species as notified by International Union for Conservation of Nature** (**IUCN) 2013 [19]. In India, it is preserved under Schedule I of Wildlife Protection Act, 1972. In the era of high concern arising worldwide in favour of conservation of wild animals, exploring an insight into the basic innate immune status of wild animals like blackbuck is warranted. Goat (*Capra hircus*) farming that contributes 8% of the gross domestic product (GDP) from livestock sector is visualized to dominate India's livestock market in the coming future. Various aspects of mechanisms and cellular responses have been widely studied in case of adaptive immune system in ruminants though the same is lacking in the innate component. In the present study, an insight has been provided into the potential ligand binding activity of innate immune component of wild versus domestic ruminants through* in silico *characterization and comparative structural analysis of the partial conglutinin encoding the neck and carbohydrate recognition domain (NCRD) of blackbuck and goat.

## 2. Materials and Methods

### 2.1. Sample Collection and RNA Isolation

Liver tissue sample of blackbuck was obtained from a carcass during necropsy examination at postmortem house, Indian Veterinary Research Institute (IVRI), Izatnagar, and goat liver sample was collected from a local abattoir. Both tissue samples were brought to the laboratory in an aseptic manner under proper cold conditions for further processing. In each case, 1 mL Trizol reagent (Life Technologies, New York, NY, USA) was added to 100–120 mg tissue and the tissue samples were homogenized using tissue homogenizer. Total RNA was isolated as per manufacturer's instructions and stored in RNase free water at −20°C. RNA absorbance was determined at 260 and 280 nm to determine quantity and ensure integrity of extracted RNA in both species.

### 2.2. cDNA Synthesis

cDNA was synthesized from respective total RNA using M-MuLV reverse transcriptase (Fermentas, USA) and oligo-dT primers (Promega, Madison, WI). A 25 *μ*L reaction mixture consisting of 5 *μ*L total RNA (1–5 *μ*g/*μ*L), 1 *μ*L oligo-dT primer (0.5 mg/mL), 1 *μ*L of RNase inhibitor (40 U/mL), 2 *μ*L of 10 mM dNTP mix, 2 *μ*L of DTT, 4 *μ*L of 5x reverse transcriptase buffer, 2 *μ*L of reverse transcriptase enzyme (5 U/*μ*L), and 6 *μ*L of nuclease-free water was prepared. The mixture was incubated at 37°C for 60 min followed by heating the reaction mixture at 70°C for 10 min to inactivate the reverse transcriptase. The synthesized cDNA of respective species was quantified using spectrophotometer (Nanodrop, USA) and stored at −20°C till use.

### 2.3. Amplification of Genes Encoding NCR Domain of Goat and Blackbuck Conglutinin

Gene encoding NCRD of conglutinin was amplified from cDNA with forward primer 5′-GGCTCGAGGGGGAGAGTGGGCTTGCAGA-3′ and reverse primer 5′-GGGAATTCTCAAAACTCGCAGATCACAA-3′ established for bovine conglutinin [20]. PCR was performed using proofreading Pfu Ultra II fusion HS DNA polymerase (Stratagene, USA). The 50 *μ*L PCR reaction mixture was prepared with 1.0 *μ*L of each the forward and reverse primers (50 pmol), 2.0 *μ*L Template cDNA, 1.0 *μ*L dNTP mix (25 mM), 5.0 *μ*L 10x reaction buffer, and 1.0 *μ*L Pfu polymerase, and final volume was made up to 50 *μ*L with nuclease-free PCR grade water. Reaction conditions were initial denaturation at 95°C for 5 min, followed by 35 repeated cycles of denaturation at 95°C for 45 sec, annealing at 58°C for 1 min, and final extension at 72°C for 5 min. The amplified products were analyzed by running 1% agarose gel electrophoresis along with the 100 bp plus DNA ladder and the ethidium bromide stained gel was visualized in gel documentation system.

### 2.4. Cloning and Characterization

The obtained PCR amplicon of each species was eluted from the gel using QIAGEN Gel extraction kit as per the manufacturer's instructions. Amplicon was ligated to pJET1.2 blunt end cloning vector (MBI, Fermentas, USA). The ligation reaction mixtures were prepared with 10.0 *μ*L 2x Ligation buffer, Insert (Purified PCR product) 3.0 *μ*L, (insert: vector molar ratio 3 : 1 was found to give optimum ligation efficiency), 1 *μ*L pJET-blunt end cloning vector (50 ng/*μ*L), and 1.0 *μ*L T4 DNA Ligase [3 U/*μ*L]. The final volume was adjusted to 20 *μ*L with nuclease-free water. The ligation was carried out at 22°C for 30 min and the product was transformed into* E. coli *DH5*α* competent cells as per the TSS protocol [21] and plated onto LB agar containing ampicillin (100 *μ*g/mL). The plates were incubated at 37°C overnight. Discrete colonies were selected from both plates and inoculated to LB broth containing ampicillin (100 *μ*g/mL) and tubes were incubated at 37°C overnight under constant shaking at 200 rpm. From the overnight grown cultures, plasmids were isolated using QIAGEN Plasmid isolation kit as per manufacturer's guidelines.

The plasmids of both species were characterized by PCR using gene specific primers as mentioned above and restriction digestion by enzyme* Pst *I (MBI Fermentas, Maryland). Restriction digestion was carried out using 3 *μ*L plasmid DNA, 2 *μ*L 10x RE buffer, and 1 *μ*L* Pst *I (10 U/*μ*L), and final volume was made up to 20 *μ*L with nuclease-free water followed by overnight incubation at 37°C. The products were resolved in 2% agarose gel electrophoresis stained with ethidium bromide and the gel was visualized in gel documentation system.

### 2.5. Sequencing and Analysis

The recombinant plasmids of both species were sequenced at First Base Laboratories Sdn Bhd Selangor, Malaysia. The obtained sequences encoding NCR domain of conglutinin were confirmed by BLAST analysis at NCBI and then submitted to Genbank. Nucleotide and predicted amino acid sequences were further compared with sequences of other domestic and wild ruminants available at NCBI Genbank, using DNAstar and MEGA5.2 softwares. Evolutionary relationship and phylogenetic variation were studied by alignments with other sequences in Mega 5.0.2 software [22]. Secondary structure and domain analysis were carried out with SMART [23] (http://smart.embl-heidelberg.de/), TMHMM [24] (http://www.cbs.dtu.dk/service/TMHMM/), and PROSITE [25] (http://www.expasy.ch/prosite), whereas quaternary structures were predicted from the deduced amino acid sequences using SWISS MODEL ProtParam [26] and PHYRE2 software [27, 28] (Protein Homology/analog Y Recognition Engine; www.sbg.bio.ic.ac.uk/phyre2). The N-glycosylation sites were predicted using HIV sequence database (www.hiv.lanl.gov) and other possible postglycosylation and phosphorylation sites were investigated with Expasy database studies (http://www.expasy.ch/prosite), whereas the expected ligand binding sites were analyzed in PREDICT PROTEIN [29] (http://www.predictprotein.org/).

## 3. Results

The quantity and integrity of extracted total RNA from both goat and blackbuck liver were estimated by measuring the RNA absorbance at 260 and 280 nm. The ratio was found to be >1.8 in both cases indicating good quality of the extracted RNA in terms of both the purity and the quantity and it was quite sufficient for the cDNA synthesis. Nearly 500 bp amplicons were obtained from PCR amplification of the cDNA with gene specific primers encoding neck and carbohydrate recognition domain (NCRD) of both species (Figure 1). The amplicons were purified, cloned, and characterized by restriction analysis and sequencing.* Pst* I restriction enzyme was used for the confirmation of two recombinant plasmids from both goat (pJET-GCGN) and blackbuck (pJET-BBCGN). Three fragments of 220 bp, 406 bp, and 2.8 kbp were obtained in restriction digestion of plasmids pJET-GCGN, whereas plasmids pJET-BBCGN upon* Pst* I digestion yielded 261 bp, 566 bp, and 2.6 kbp fragments due to reverse orientation (Figure 2). Characterized recombinant plasmids were sequenced and analyzed* in silico. *These sequences have been assigned NCBI GenBank accession numbers KC505182 and KC505183 for blackbuck and goat, respectively. Sequence analysis revealed that the partial cDNA encoding the NCR domain of both blackbuck and goat conglutinin consisted of 497 bp with an ORF of 488 bp encoding a polypeptide of 162 amino acids having 17.6 kDa molecular weight.

Predicted protein sequence of partial goat conglutinin by EditSeq (DNAstar) revealed the presence of 14 strongly basic (+) (K,R), 19 strongly acidic (−) (D,E), 54 hydrophobic (A,I,L,F,W,V), and 52 polar (N,C,Q,S,T,Y) amino acids with isoelectric point at 4.980 and −4.858 charge at pH 7.0. Gene sequence was found to comprise of 26.54% A (129), 27.57% G (134), 19.75% T (96), 26.13% C (127), 46.30% A+T (225), and 53.70% C+G (261). Similarly, predicted protein sequence of partial blackbuck conglutinin contained 19 strongly basic (+) amino acids (K,R), 22 strongly acidic (−) amino acids (D,E), 50 hydrophobic amino acids (A,I,L,F,W,V), and 47 polar amino acids (N,C,Q,S,T,Y), isoelectric point at 5.505 with −2.853 charge at pH 7.0. Gene sequence contained 28.19% A, 29.01% G, 19.55% T, 23.25% C, 47.74% A+T, and 52.26% C+G.

For comparative sequence analysis, partial conglutinin nucleotide sequences of other ruminants like cattle (UO6860.1), buffalo (HQ330990), nilgai (HQ330991), and sheep (JQ692170) along with the sequences of three bovine collectins like CL-43 (NM_001002237.1), CL-46 (NM_001001856.1), and SP-D (NM_181026.2) were retrieved from the GenBank. For possible three dimensional structural analysis, amino acid sequences of recombinant human SP-D (rhSP-D) and recombinant rat SP-A (rrSP-A) were obtained from protein data bank (PDB) with accession numbers P35247 and U43092, respectively. Both sequences of goat and blackbuck were aligned with retrieved sequences using Clustal (W) method of Mega 5.2 software and percent identity and divergence were determined (Figure 3). This cross-species alignment of goat partial cDNA revealed percentage similarity up to validate values of 92.4%, 93.4%, 93.4%, 98.2%, 93.6%, 81.1%, 89.5%, 77.1%, 64.9%, and 49.2% with those of cattle, buffalo, nilgai, sheep, blackbuck, cattle CL-43, cattle CL-46, cattle SP-D, rhSP-D, and rrSP-D, respectively, whereas blackbuck partial cDNA was found to display 95.7%, 99.8%, 99.8%, 93.2%, 93.6%, 82.3%, 90.1%, 76.8%, 65.8%, and 49.2% similarity with cattle, buffalo, nilgai, goat, sheep, cattle CL-43, cattle CL-46, cattle SP-D, rhSP-D, and rrSP-D, respectively, at nucleotide level. Similar alignment of predicted amino acid sequences (Figure 4) of conglutinin encoding the NCR domain displayed 88.3%, 88.9%, 88.9%, 98.1%, 88.9%, 70.2, 80.9, 64.8, 62.9, and 32.1 similarity of goat with those of cattle, buffalo, nilgai, sheep, blackbuck, cattle CL-43, cattle CL-46, cattle SP-D, rhSP-D, and rrSP-D, respectively, whereas those of blackbuck exhibited 96.3%, 99.8%, 99.8%, 88.9%, 88.9%, 73.3%, 82.7%, 66.4%, 61.6%, and 33.3% similarity with cattle, buffalo, nilgai, goat, sheep, cattle CL-43, cattle CL-46, cattle SP-D, rhSP-D, and rrSP-D, respectively.

Nucleotide phylogram revealed an independent cluster for wild ruminants like buffalo, nilgai, and blackbuck from those of domestic ruminants like cattle, sheep, and goat apart from other collectins. Further among the ruminants, small ruminants have created an independent cluster separately from large ruminants while descending from a common ancestor. Similar phylogenetic divergence was also observed at the level of predicted amino acid sequences as indicated in the phylogram (Figure 5). The presence of four cysteine amino acids at positions 65, 137, 151, and 159 was found to be conserved in conglutinin of all the species and other lectins indicating its specific role in forming the active dodecameric structure of the protein.

Structural prediction from the amino acid sequences deduced from the partial cDNA sequences based on PROSITE and SMART analysis tools (Figure 6) revealed the presence of a coiled-coil-like region extending from 6 to 28 amino acids and a C-type lectin domain (CLECT) from 37 to 160 amino acids consisting of the conserved signature sequence of CVEISPEGQWNDIPCSKQLLVIC between 137 and 159 residues. Further, four conserved cysteine residues present in the C-type lectin domain (CTLD) were found to form two intradomain disulphide bonds between 65–159 and 137–151 residues. The PHYRE automatic fold recognition analysis tool was used for modeling the 161 residues of the predicted polypeptide with 100% confidence to deduce the predicted secondary structure and the polypeptide was found to consist of 3 *α*-helices (4–31, 58–68, and 78–89) and 6 *β*-sheets (42–52, 71–75, 95–101, 107–110, 138–148, and 155–161) (Figure 7). The same result was also obtained by the SWISS MODEL ProtParam analysis for secondary structure folding pattern. TMHMM prediction denied the presence of any hydrophobic transmembrane helical region suggesting extracellular localization of the protein. PROSITE analysis of the deduced amino acid sequence revealed the only predicted N-glycosylation site to be at Asp-127 and the possible acetylation site at Ser-3. Potent phosphorylation sites were deduced to be at Thr-16, Ser-57, Ser77, Ser98, and Tyr-96 in case of conglutinin. No sites were found for myristoylation whereas Trp-121 was found to be the site for mannosylation.

## 4. Discussion

Immune system plays a vital role in the survival of vertebrates regularly confronted with thousands of pathogens varying from micro level viral and bacterial particles to metazoans like helminthes. Among the two wings of immune system, adaptive one helps in processing, presentation, and destruction of foreign pathogens, whereas innate one helps in recognition of PAMP through PRR. Research in the area exploring various aspects of immune system in ruminants is gaining pace; still, little information exists in wild counterparts. In this regard, the present piece of work reporting cloning and characterization of partial cds in goat and blackbuck adds further information to the innate immune status of ruminants.

In the present study, the amplified cDNA encoding the NCR domain of conglutinin in goat and blackbuck was found to be consisting of 497 bp with an ORF of 488 bp that encodes a polypeptide of 161 amino acids lacking the N terminal cysteine-rich noncollagenous domain. The positive amplification from the liver tissue samples strengthens the concept that liver is the main site of synthesis of conglutinin as was reported by Suzuki et al. [1], Liou et al. [2], and Lu et al. [4] in case of cattle; however, it is not confined to bovines. Though, northern-blot analysis on total RNA purified from cattle and sheep lungs revealed weak signal at 1.8 kb possibly due to cross-hybridization with SP-D mRNA [4], yet the expression of conglutinin in wild and domestic ruminant lungs has not been reported so far. The restriction digestion patterns of recombinant plasmids (pJET-GCGN and pJET-BBCGN) with* Pst *I restriction enzyme were found to be approximately similar with those obtained for partial cDNA sequences of cattle, buffalo, nilgai, and sheep indicating conservation of the restriction site in partial conglutinin of these ruminants [30]. Conservation of the four cysteine residues (Cys-65, 137, 151, and 159) with presence of three residues in signature sequence supports the findings of Hoppe [31] for lectin domains. The three cysteine residues (Cys-135, 151, 159) in the signature sequence play an important role in folding pattern of CRD stabilizing the conformation through exposure of specific domain [31]. Posttranslational modification patterns were also found to be conserved in all the species indicating similar type of interaction between the amino acid residues in establishing three *α*-helices and six *β*-sheets. Asp-127 was found to be the most potent N-glycosylation site and Ser-3 was found as the site for acetylation. Tyr-121 was predicted as the site for mannosylation whereas no sites were observed for myristoylation purpose. Expected sites for phosphorylation include Thr-16. Ser-57, Ser-77, Ser-98, and Tyr-96, and Lys at the positions 33, 50, 56, 82, and 92 can be assessed as the sites for glycation through its epsilon amino group. Although the sites on the protein are predicted in this report, yet the presence of actual posttranslational modifications at all these sites is yet to be established.

High resolution X-ray crystallographic structure of a recombinant fragment of human SP-D from residues 179–355 (rhSP-D; [32, 33]) and rat SP-A from residues 81–228 (rrSP-A; [34]) has been reported in both native and ligand-bound form. Comparative study with both of the above sequences has paved a way for exploring the subtle variation in geometry of CRDs with special reference to potential saccharide affinity.

The conserved* cis*-Pro-235, Lys-246, and Lys-229 and the asymmetric Tyr-228 in rhSP-D as reported by Shrive et al. [33] corresponding to positions-39, 50, 33, and 32 in partial conglutinin of all the six species have specific role in neck to CRD transition, stabilizing the internal interactions of trimer. Further residues including His-220, Gln-227, Lys-229, Lys-230, and Glu-242 in rhSP-D [33] are conserved in conglutinin corresponding to positions-24, 31, 33, 34, and 46, respectively, that have a role in connecting the central pore at the bottom of the funnel created by the three CRDs with the cleft formed by the CRD and the neck peptide. It confirms the similarity of the conglutinin molecule with that of SP-D in formation of dodecameric cruciform structure. Glu-232 in the rhSP-D trimer that forms a charged surface at the bottom of CRD funnel and binds to calcium ion has vital role in recognition of LPS, phospholipid, and immune cells [32, 33, 35]. It is replaced by Val-36 in partial conglutinin that may contribute towards the variation in flexibility and ligand binding activity. Three calcium ions are required to be coordinated with the CRD region for the functional saccharide (glucose, mannose) binding activity as reported by Shrive et al. [33]. The Ca-binding loop in rhSP-D formed by the residues Glu-321, Asn-323, Glu-329, Asn-341, and Asp-342 corresponding to residues 125, 127, 135, 147, and 148, respectively, is also conserved in CR domain of predicted partial conglutinin. This finding is in accordance with the mandatory requirement of calcium for ligand binding in case of conglutinin like those of other collectin groups of proteins as revealed by Iobst et al. [36].

Arginine residue plays an important role in ligand binding functional activity as reported by the X-ray analysis of lectin [37]. In this aspect, the presence of Arg-14 and Arg-66 in cattle, buffalo, nilgai, and blackbuck replacing Glu-14 and Thr-66 of sheep and goat in the coiled and lectin domain, respectively, may explain the variation in strength of ligand binding activity. Further, Allen et al. [38] have reported through gene deletion mutant studies that in human surfactant protein-D, Arg-343 is the key element in discrimination between glucose and N-acetylglucosamine ligands. Replacement by Val-149 in cattle, buffalo, nilgai, and blackbuck and by Ile-149 in sheep and goat partial conglutinin may contribute towards* in vitro* saccharide affinity studies which need to be explored experimentally. Similarly, presence of hydroxyl and carbonyl side chain in the CR domain is found to act as the Ca^2+^ binding sites during recognition of PAMP on microbial surface. So, the presence of Ser-78 in cattle; Glu-78 in buffalo and nilgai; Glu-82 in cattle, buffalo, and nilgai replacing the hydrophobic Ala-78 and Lys-82 in sheep and goat in CR domain may explain the discrepancies in potential functional activity that is yet to be established.

A difference in the three-dimensional quarternary structure of conglutinin of goat, sheep, and cattle from that of buffalo, nilgai, and blackbuck has been observed, suggesting thereby that there may be a difference in the ligand binding efficiency and resulting antimicrobial activity among the wild and domestic ruminants. The degree of subunit oligomerization probably affects the recognition of and binding strength to the carbohydrate ligands on the surface of pathogens [39]. In this regard, 4–31 coiled coil region bearing a Cys-65 plays the center stage in initiating the process as indicated by diffraction studies of rhSP-D and rrSP-A [31–33]. The existing variation in the SWISS MODEL predicted quaternary structure can be attributed to the presence of hydrophobic Ala-52 at neck-CRD interface in sheep, goat, and cattle identical to that of SP-D, whereas in buffalo, nilgai, and blackbuck, replacement by Thr-52 might have some structural importance that needs to be discovered through high resolution X-ray diffraction studies. The tertiary level difference in folding pattern of conglutinin in wild versus domestic ruminants may have specific role in their ligand binding and functional activity contributing towards innate immune response that needs to be explored further.

Wild animals surviving in a hoarse environment while constantly getting exposed to various pathogens are supposed to possess strong innate immunity as compared to the domestic animals [40]. Reports are available regarding characterization of innate immune markers like TLR-3 [41] and TLR-2 [42] in water buffalo and nilgai; IFN-alpha [43] in goat and blackbuck; IL-2 [44] and IL-18 [45] in nilgai. The present piece of work is the first report of cloning, characterization, and* in silico* sequence analysis of partial cds of conglutinin in goat and blackbuck. Software-based homology, phylogeny, and structural analysis revealed that blackbuck conglutinin is similar to that of nilgai and buffalo, whereas goat conglutinin is closer to that of sheep. Comparative study with SP-D reflects the structural variation of wild ruminants from domestic ones that paves a way for future studies on functional ligand binding activities through various experimental evidences.

## Figures and Tables

**Figure 1:** PCR amplification of cDNA encoding conglutinin NCR domain (Lane M: 100 bp plus DNA ladder, (a) Lane 1: goat PCR amplicon of ~500 bp, and (b) Lane 1: blackbuck PCR amplicon of ~500 bp).

**Figure 2:** Restriction digestion of recombinant plasmids by* Pst *I restriction digestion (Lane M: 100 bp plus DNA ladder, (a) insert release of 220 bp, 406 bp, and 2.8 kb from goat recombinant plasmids (pJET-GCGN) Lane 1-2, and (b) insert release of 261 bp, 566 bp, and 2.6 kb from blackbuck recombinant plasmids (pJET-BBCGN) Lane 1-2).

**Figure 3:** Alignment of nucleotide sequences of goat and blackbuck conglutinin NCRD with sequences of other ruminants (cattle, buffalo, sheep, and nilgai) and collectins (cattle collectin-43, cattle collectin-46, cattle surfactant protein-D, recombinant human surfactant protein-D (rhSP-D), and recombinant rat surfactant protein-A (rrSP-A)). Identity of the sequences is indicated by dots and the differences by the corresponding nucleotide symbols. Gaps introduced for optimal alignment are indicated by dashes. The GenBank accessions are given in parentheses.

**Figure 4:** Alignment of predicted amino acid sequences of goat and blackbuck conglutinin NCRD with other wild and domestic ruminants (cattle, buffalo, sheep, and nilgai) and collectins (cattle collectin-43, cattle collectin-46, cattle surfactant protein-D, recombinant human surfactant protein D (rhSP-D), and recombinant rat surfactant protein A (rrSP-A)). Identity of the sequences is indicated by dots and the differences by corresponding one letter symbol of amino acids. Gaps introduced for optimal alignment are indicated by dashes. Four conserved cysteine residues are indicated by vertical (green) boxes. Predicted regions of secondary structures are indicated by horizontal (blue) boxes (A1-alpha helical region-1, A2-alpha helical region-2, A3-alpha helical region-3, B1-beta sheet region-1, B2-beta sheet region-2, B3-beta sheet region-3, B4-beta sheet region-4, B5-beta sheet region-5, and B6-beta sheet region-6). Three regions, collagen triplet, coiled neck, and lectin domain, are distinctly demarcated by the sequences confined within the red arrow marks. The signature sequences within lectin domain are indicated by red horizontal box.

**Figure 5:** Phylogenetic relationship between the predicted amino acid sequences for the NCR domain of conglutinin from different species (cattle, buffalo, nilgai, blackbuck, sheep, and goat) and collectins (cattle collectin-43, cattle collectin-46, cattle surfactant protein-D, recombinant human surfactant protein D (rhSP-D), and recombinant rat surfactant protein A (rrSP-A)) using Mega version 5.1 Clustal W method. Numbers outside the branches indicate the bootstrap values obtained using 1,000 replicates and values above 50% are shown. The scale bar at the bottom measures the amino acid substitutions per site for a unit branch length.

**Figure 6:** Phyre2 software predicted secondary structure from partial conglutinin amino acid sequences, (a) blackbuck and (b) goat.

**Figure 7:** (a) SWISS MODEL predicted structure of NCRD region of conglutinin of various wild and domestic ruminant species (cattle, buffalo, nilgai, blackbuck, sheep, and goat). (b) SWISS MODEL predicted and PDB modeled structure of SP-D.
